The article "Whole-exome sequencing analysis of amniotic fluid cells in 5 pregnant women with thalassemia: Case report" was published in 2022. Journal: Medicine (Baltimore).

# Whole-exome sequencing analysis of amniotic fluid cells in 5 pregnant women with thalassemia: Case report

**DOI:** 10.1097/MD.0000000000031645

**Published:** 2022-11-25

**Authors:** Wei Zhang, Xiaokang Li, Xiaoxia Wu, Xin Huang, Xiao Zhang, Yi Lu, Jianmin Niu, Jian Zhang

**Affiliations:** a Shenzhen Key Laboratory of Cardiovascular Health and Precision Medicine, Southern University of Science and Technology, Shenzhen, Guangdong, China; b School of Medicine, Southern University of Science and Technology, Shenzhen, Guangdong, China; c School of Public Health and Emergency Management, Southern University of Science and Technology, Shenzhen, Guangdong, China; d Shenzhen Jinxin Medical Technology Innovation Center, Co., Ltd., Shenzhen, Guangdong, China; e Affiliated Shenzhen Maternity & Child Healthcare Hospital, Southern Medical University, Shenzhen, Guangdong, China; f Guangdong Provincial Key Laboratory of Cell Microenvironment and Disease Research, Shenzhen, Guangdong, China.

**Keywords:** α-thalassemia, β-thalassemia, case report, amniocyte fluid cell, whole-exome sequencing

## Abstract

While thalassemia is a monogenic disease that is relatively common worldwide, there is no recognized radical cure for thalassemia in current medical practice. Prenatal diagnosis is the most important contribution to thalassemia prevention, but due to its technical limitations, rare thalassemia mutations cannot be detected; and the birth of thalassemic babies cannot be completely circumvented. Whole-exome sequencing can, however, compensate for this shortcoming.

**Patient concerns:**

We report the results of whole exon sequencing of amniotic cells in 5 pregnant women with thalassemia.

**Diagnosis:**

Prenatal diagnosis revealed that 4 of them were α thalassemia carriers and 1 of them was β thalassemia carrier.

**Interventions and Outcomes:**

We collected amniotic fluid of 5 pregnant women (age range: 25–27 years, Mean ± SD: 28 ± 1.8) with thalassemia. The gestational ages ranged between 16 and 19 weeks. The cells were separated from the amniotic fluid and passaged until a sufficient number of cells were obtained for exome sequencing. We therefore employed whole-exome sequencing of amniotic fluid cells from thalassemic carriers to validate prenatal diagnostic results and to identify novel mutation sites. We found that 4 of 5 samples are SEA which is consistent with the clinical prenatal diagnosis. However, 2 of 5 samples were point mutations in the HBB gene, and were thus different from the clinical prenatal diagnosis.

**Conclusion:**

The identifications from this study showed that prenatal diagnosis has limitations. Whole-exome sequencing can compensate for this shortcoming. And this study would add new insights into understanding of molecular mechanisms in thalassemia.

## 1. Introduction

The original term “thalassemia” denoted a Mediterranean anemia, as most of the early cases were found in coastal regions of the Mediterranean Sea. However, there are many different types with respect to clinical symptoms, with only anemia and hemolysis as common signs. Therefore, thalassemia is actually a group of disorders, and its etiology entails a deletion or mutation of a globin gene that results in 1 or more defects in globin peptide-chain synthesis. This defect results in a severe imbalance in the ratio of α-globin to β-globin in the hemoglobin molecule, and unbalanced synthetic rates in α- and β-globins then generate anemia.^[1–3]^ Although routine clinical treatments include blood transfusion, iron chelation, and splenectomy, hematopoietic stem cell transplantation has shown to be the most effective method for curing thalassemia.^[4–6]^ As allogeneic hematopoietic stem cell transplantation is limited to patients with a human leukocyte antigen-syngeneic donor, matching remains difficult; and sources of bone marrow (hematopoietic stem cells) are rare—with potential graft-versus-host disease severely limiting the promotion of this treatment.^[4]^ γ-globin gene activation is now 1 of the most effective treatments for β-thalassemia: drugs are used to stimulate the effective expression of the γ-globin gene that is repressed after birth, and this improves the imbalance in α- and non-α-globin synthesis and increases fetal hemoglobin synthesis to reduce hemolysis and alleviate anemia.^[7,8]^ While numerous drugs can induce γ-globin expression or promote fetal hemoglobin synthesis, many possess deficiencies such as poor efficacy, severely toxic side-effects, and a short half-life.^[9,10]^ Prenatal diagnosis is therefore an effective measure used to prevent the birth of severely thalassemic babies. Invasive prenatal diagnostic methods principally involve the collection of fetal genetic material from the chorion, amniotic fluid, and umbilical cord blood for laboratory testing; and samples that exhibit positive screening results are then used for further genetic analysis and diagnosis. However, this methodology usually only detects common mutation sites in the α- and β-globin gene clusters, resulting in an inability to distinguish rare thalassemic mutations. As exome sequencing can compensate for this shortcoming, we employed this modality to sequence amniotic fluid cells from thalassemia carriers; and this allowed us to validate prenatal diagnostic results and to uncover novel mutation sites.

## 2. Case report

We collected amniotic fluid from 5 pregnant women who were thalassemia carriers at gestational ages between 16 and 19 weeks (i.e., mid-second trimester) (Table 1). Hypochromic and microcytic red blood cells and target cells were shown in the peripheral blood smear of patients with thalassemia (Fig. 1A). We used gradient centrifugation to isolate fetal fibroblasts for in vitro culture. After 14 days of culturing fetal fibroblasts to allow proliferation (Fig. 1B), we extracted genomic DNA from the cells for Whole-exome sequencing (WES). Of the 5 samples, the clinical prenatal diagnostic results showed 4 amniotic fluid samples from Southeast Asian deletion (--SEA) α-thalassemia carriers and 1 from a CD27-28 (+C, frameshift mutation) β-thalassemia carrier (Table 1).

**Table 1:** Clinical prenatal diagnosis and gene type of the 5 samples.

Sample	Gestational age (wks)	Clinical diagnosis	Gene type
N1	16^+5^	α thalassemia heterozygote	--SEA
N2	18^+4^	α thalassemia heterozygote	--SEA
N3	16^+6^	α thalassemia heterozygote	--SEA
N4	16^+^	α thalassemia heterozygote	--SEA
N5	18^+4^	β thalassemia heterozygote	CD27-28 (+C)

**Figure 1.** Pictures of blood smear and amniotic fluid cells. A: The blood smear of normal person (left) and thalassemia (right). B: Photomicrographs of amniotic fluid cells on day 0 and day14.

By exploiting the East Asian 1000 Genomes database, we compared the normal copy number of chromosomal genes in the HGNC database to obtain the copy number variation (CNV) for genes on every chromosome (data were not shown), and noted that most α-thalassemia cases were due to fragment deletion. As we observed numerous CNVs for the α-globin gene, we screened for globin-gene copy number in our exome-sequencing data. We determined that the copy number for the α-globin genes HBA1 and HBA2 on chromosome 16 in 4 samples (N1, N2, N3, N4) was 1, and that there was copy number loss (the normal copy number for α-globin genes HBA1 and HBA2 is 2). Only the N5 sample manifested a copy number of 2 for HBA1 and HBA2 (Fig. 2). These results were consistent with the clinical prenatal diagnosis that the N1, N2, N3, and N4 samples were from --SEA α-thalassemia carriers (Table 2).

**Table 2:** Clinical prenatal diagnosis and whole-exon sequencing results of the 5 samples.

Sample	Diagnostic genotype	Whole-exome sequencing
N1	--SEA	Both HBA1 and HBA2 only have 1 copy/HBB gene mutation (rs10768683: G > C)
N2	--SEA	Both HBA1 and HBA2 only have 1 copy
N3	--SEA	Both HBA1 and HBA2 only have 1 copy
N4	--SEA	Both HBA1 and HBA2 only have 1 copy
N5	CD27-28 (+C)	HBB gene mutation (rs10768683: G > C)

**Figure 2.** Statistical analysis of HBA1 and HBA2 gene copy number in the 5 samples. A: HBA1 gene copy number in the 5 samples. B: HBA2 gene copy number in the 5 samples. The yellow dots represent insert (INS), blue dots represent delete (DEL), and red dots represent normal.

A majority of β-thalassemia cases are due to point mutations, and, therefore, single-nucleotide polymorphism (SNP) and small insertion and deletion (InDel) mutation annotations can be used for screening. The β-globin (HBB) gene is located on chromosome 11, and we located a point mutation (rs10768683: G > C) on the β-globin gene (ENSG00000244734) in the N1 and N5 samples; these were non-synonymous SNP mutations that resulted in a single amino acid substitution (A-P) (Fig. 3). This outcome was thus significantly different from the clinical prenatal diagnosis that revealed that only the N5 sample reflected a CD27-28 (+C, frameshift mutation) mutation in the HBB gene (Table 2).

**Figure 3.** β-globin-mutation screening. A: HBB gene-mutation sites in N1 and N5 samples. WT, normal human gene type; MUT, mutation; B, β-globin point mutation (G > C) in N1 and N5 samples.

There are abundant mutation sites in the human genome, and some mutations are extremely common and proven not to alter normal human survival rates. However, some mutations are highly correlated with human disease, and we applied GATK software for statistical analysis of SNP and InDel mutations^[11]^ (Table 3). In order to identify significant disease mutations, we used ANNOVAR software for annotation analysis of the detected SNP and InDel mutations combined with external databases to confirm the genome location, mutation frequency, protein harmfulness, genotype heterozygosity, and functional pathway information.^[12]^ GO-enrichment analysis was executed on the common mutation sites in the 5 samples and 26 terms were significantly enriched based upon the false-discovery rate-corrected *P* value (i.e., *q* value) of .05 as the upper limit. The Gene Ontology (GO) terms included plasma membrane, actin cytoskeleton, extracellular matrix structural constituent, calcium ion binding, and transmembrane signaling receptor activity (Fig. 4). When we used Kyoto Encyclopedia of Genes and Genomes-enrichment analysis for the common mutation sites, we noted 13 signaling pathways as significantly enriched—including sugar metabolism, β-alanine metabolism, ECM receptor interaction, and complement and coagulation cascades (Fig. 5).

**Table 3:** SNP-InDel statistics of the 5 samples.

Sample	Number of SNPs	Number of InDels
N1	47347	4053
N2	47792	4097
N3	47869	4068
N4	47697	3969
N5	48190	4048

SNP = single-nucleotide polymorphism.

**Figure 4.** The significantly enriched biological functions of the common SNP and Indel using GO are illustrated in bar chart. GO = Gene Ontology, SNP = single-nucleotide polymorphism.

**Figure 5.** The significantly enriched pathways using KEGG pathway analysis are illustrated in the dot plots. Rich factor refers to the proportion of DMGs belonging to a specific term, node size (gene number) refers to the number of SNPs and Indels within each term, and node color indicates the level of significance (−log10 *P* value). DMGs = differentially methylated genes, KEGG = Kyoto Encyclopedia of Genes and Genomes.

## 3. Discussion

Thalassemia is a monogenic disorder that exhibits a high global incidence. Even though improvements have been made in thalassemia advocacy and prenatal diagnosis, there remain many patients who are afflicted but not yet identified. We performed exome sequencing amniotic fluid cells from 5 pregnant women who were thalassemia carriers, and CNV results showed that α-globin gene-copy loss was present in 4 samples, which was congruent with clinical prenatal results of --SEA α-thalassemia-carrier status in 4 corresponding samples. SNP and InDel mutation annotation screening, however, revealed that non-synonymous mutation in the HBB gene was found in the N1 and N5 samples, which differed significantly from the clinical prenatal results that showed that only the N5 sample contained a CD27-28 (+C, frameshift mutation) in the HBB gene. These data show that exome sequencing can complement the shortcomings of prenatal clinical diagnosis, and that it is an effective tool for identifying novel thalassemia-mutation sites.

GO-enrichment analysis of the mutated genes showed that 26 terms were significantly enriched, including plasma membrane, actin cytoskeleton, and extracellular matrix structural constituent. Athanasiou et al employed micropipette aspiration to measure the elastic shear modulus in erythrocytes from both a thalassemic mouse model and from patients with thalassemia, and demonstrated that their erythrocyte stiffness was significantly greater than in normal erythrocytes.^[13]^ Investigators reported that a diminution in erythrocyte deformability and membrane stability induced the destruction of erythrocytes as they passed through the medullary cavity, splenic sinusoids, and capillary network; and that it shortened both erythrocyte lifespan in blood and an affected individual’s lifespan.^[14]^ We subsequently carried out Kyoto Encyclopedia of Genes and Genomes-enrichment analysis on the mutated genes, and ascertained that 13 signaling pathways were significantly enriched—including sugar metabolism and complement and coagulation cascades. Chen et al also demonstrated that thalassemia was correlated with complications of diabetes mellitus, as type 2 diabetics exhibited higher levels of serum ferritin relative to non-diabetic individuals.^[15]^ Luo Y. et al conducted a study on 79 moderately thalassemic patients (114 of whom had HbH and 18 with HbE/β), and reported that 33 were hypoglycemic, 25 showed impaired glucose tolerance, and 4 manifested diabetes. Impaired glucose tolerance in symptomatic diabetes mellitus was substantiated for thalassemic patients.^[16]^ An excess of deformed globin chains in thalassemic erythrocytes are deposited on the erythrocyte membrane, leading to membrane protein aggregation and binding to autoantibodies and complement, and this in turn promotes the rapid clearance of erythrocytes in the circulation.^[17]^ Abnormalities of the innate immune system associated with thalassemia were reported including reduced absorption and phagocytic ability of polymorphonuclear neutrophils, and altered intracellular metabolic processes.^[18,19]^ Complement is a part of the innate immune system which plays an essential role in defense against pathogens and intissue homeostasis.^[20]^ Hemolytic diseases are often accompanied by dysregulation and overactivation of the complement system, which may be induced by free extracellular heme.^[21–23]^ In our study, we uncovered complement-related immune abnormalities in thalassemic fetuses.

YeeHo et al used pyrosequencing to detect beta-thalassemia mutations in prenatal samples (chorionic villus biopsies and cultured and uncultured amniocytes). However, pyrosequencing has strict requirements on the concentration of DNA template, and the presence of maternal cell contamination can interfere with interpretation of results, particularly when the fetus carries the same mutation as the mother.^[24]^ Murad et al used molecular screening and direct DNA sequencing to evaluate a prenatal diagnosis of β-thalassemia by collecting 55 amniotic fluid samples in Syria.^[25]^ In another study fetal cells were isolated using micromanipulators at 8 weeks of gestation in women with high-risk pregnancies and nested polymerase chain reactions were performed.^[26]^ That study demonstrated that prenatal diagnosis of β thalassemia may be feasible at an early stage of pregnancy. In our study, we performed WES to analyze amniotic fluid cells from 5 pregnant women who were thalassemia carriers, and noted WES as an effective tool for identifying novel thalassemia-mutation sites. However, since exome sequencing requires high DNA concentrations, the process requires 10 to 14 days of cell culture in vitro; and the high sequencing costs also limit its use in clinical prenatal diagnosis. The obstetricians/gynaecologists were most concerned that ordering an expansive test could lead to overtreatment, higher cost of care and may increase parental anxiety.

## 4. Conclusion

In conclusion, we found that the use of exome sequencing enables a more comprehensive analysis of mutation sites. As the costs of sequencing fall, and bioinformatic and analytic capabilities improve，this will improve diagnostic capabilities because of improved ability to detect a wider range of genomic abnormalities, including non-coding variants, copy number changes and larger rearrangements. We will further accumulate the number of samples, in order to provide reliable evidence for improving the accuracy and sensitivity of clinical diagnosis of thalassemia.

## Author contributions

JMN, YL and JZ designed research; XKL, XH, XZ performed research; WZ, XKL, XXW analyzed data; WZ, XKL and XXW wrote the paper.

**Conceptualization:** Yi Lu, Jianmin Niu.

**Data curation:** Wei Zhang, Xiaokang Li.

**Formal analysis:** Yi Lu.

**Funding acquisition:** Jian Zhang.

**Methodology:** Xiaoxia Wu, Xin Huang.

**Software:** Xin Huang, Xiao Zhang.

**Supervision:** Jian Zhang.

**Writing – original draft:** Wei Zhang, Xiaokang Li.

**Writing – review & editing:** Yi Lu, Jianmin Niu, Jian Zhang.

## References

[1] CleggJBWeatherallDJ. Molecular basis of thalassaemia. Br Med Bull. 1976;32:262–9.78883610.1093/oxfordjournals.bmb.a071373

[2] RundDRachmilewitzE. Beta-thalassemia. N Engl J Med. 2005;353:1135–46.1616288410.1056/NEJMra050436

[3] CaoAGalanelloR. Beta-thalassemia. Genet Med. 2010;12:61–76.2009832810.1097/GIM.0b013e3181cd68ed

[4] BaroncianiDAngelucciEPotschgerU. Hemopoietic stem cell transplantation in thalassemia: a report from the European Society for Blood and Bone Marrow Transplantation Hemoglobinopathy Registry, 2000-2010. Bone Marrow Transp. 2016;51:536–41.10.1038/bmt.2015.29326752139

[5] La NasaGGiardiniCArgioluF. Unrelated donor bone marrow transplantation for thalassemia: the effect of extended haplotypes. Blood. 2002;99:4350–6.1203686110.1182/blood.v99.12.4350

[6] HongengSPakakasamaSChaisiripoomkereW. Outcome of transplantation with unrelated donor bone marrow in children with severe thalassaemia. Bone Marrow Transplant. 2004;33:377–9.1467678110.1038/sj.bmt.1704361

[7] GnanapragasamMNScarsdaleJNAmayaML. p66Alpha-MBD2 coiled-coil interaction and recruitment of Mi-2 are critical for globin gene silencing by the MBD2-NuRD complex. Proc Natl Acad Sci USA. 2011;108:7487–92.2149030110.1073/pnas.1015341108PMC3088629

[8] RuponJWWangSZGaenslerK. Methyl binding domain protein 2 mediates gamma-globin gene silencing in adult human betaYAC transgenic mice. Proc Natl Acad Sci USA. 2006;103:6617–22.1660891210.1073/pnas.0509322103PMC1458932

[9] MettanandaSFisherCAHayD. Editing an alpha-globin enhancer in primary human hematopoietic stem cells as a treatment for beta-thalassemia. Nat Commun. 2017;8:424.2887114810.1038/s41467-017-00479-7PMC5583283

[10] El-BeshlawyAEl-GhamrawyM. Recent trends in treatment of thalassemia. Blood Cells Mol Dis. 2019;76:53–8.3079216910.1016/j.bcmd.2019.01.006

[11] DePristoMABanksEPoplinR. A framework for variation discovery and genotyping using next-generation DNA sequencing data. Nat Genet. 2011;43:491–8.2147888910.1038/ng.806PMC3083463

[12] WangKLiMHakonarsonH. ANNOVAR: functional annotation of genetic variants from high-throughput sequencing data. Nucleic Acids Res. 2010;38:e164.2060168510.1093/nar/gkq603PMC2938201

[13] AthanasiouGZoubosNMissirlisY. Erythrocyte membrane deformability in patients with thalassemia syndromes. Nouv Rev Fr Hematol. 1991;33:15–20.1945820

[14] SchrierSLRachmilewitzEMohandasN. Cellular and membrane properties of alpha and beta thalassemic erythrocytes are different: implication for differences in clinical manifestations. Blood. 1989;74:2194–202.2804358

[15] ChenLLiYZhangF. Elevated serum ferritin concentration is associated with incident type 2 diabetes mellitus in a Chinese population: a prospective cohort study. Diabetes Res Clin Pract. 2018;139:155–62.2952448310.1016/j.diabres.2018.03.001

[16] LuoYBajoriaRLaiY. Prevalence of abnormal glucose homeostasis in Chinese patients with non-transfusion-dependent thalassemia. Diab Metab Syndr Obes. 2019;12:457–68.10.2147/DMSO.S194591PMC648962231114275

[17] YuanJKannanRShinarE. Isolation, characterization, and immunoprecipitation studies of immune complexes from membranes of beta-thalassemic erythrocytes. Blood. 1992;79:3007–13.1586745

[18] LawsonSERobertsIAGAmroliaP. Bone marrow transplantation for beta—thalassaemia major: the UK experience in two paediatric centres. Br J Haematol. 2003;120:289–95.1254248910.1046/j.1365-2141.2003.04065.x

[19] SinsJW. Early occurrence of red blood cell alloimmunization in patients with sickle cell disease. Am J Hematol. 2016;91:763–9.2710271910.1002/ajh.24397

[20] RicklinDHajishengallisGYangK. Complement: a key system for immune surveillance and homeostasis. Nat Immunol. 2010;11:785–97.2072058610.1038/ni.1923PMC2924908

[21] MoldCTameriusJDPhillipsG. Complement activation during painful crisis in sickle cell anemia. Clin Immunol Immunopathol. 1995;76:314–20.755445410.1006/clin.1995.1131

[22] BiryukovSStouteJA. Complement activation in malaria: friend or foe? Trends Mol Med. 2014;20:293–301.2450827510.1016/j.molmed.2014.01.001

[23] LubkaT. Heme: modulator of plasma systems in hemolytic diseases. Trends Mol Med. 2016;22:200–13.2687544910.1016/j.molmed.2016.01.004

[24] YeeHoS. Rapid prenatal diagnosis of common beta-thalassemia mutations in Southeast Asia using pyrosequencing. Prenat Diagn. 2013;33:1017–22.2379414410.1002/pd.4183

[25] MuradHMoassasFJarjourR. Prenatal molecular diagnosis of β-thalassemia and sickle cell anemia in the Syrian popularion. Hemoglobin. 2014;38:390–3.2540591610.3109/03630269.2014.978455

[26] GiambonaA. Early prenatal diagnosis of Hb Lepore Boston-Washington and β-thalassemia on fetal celomatic DNA. Int J Lab Hematol. 2022;44:796–802.3533343310.1111/ijlh.13837

